# Optimization Simulation of Dance Technical Movements and Music Matching Based on Multifeature Fusion

**DOI:** 10.1155/2022/8679748

**Published:** 2022-06-08

**Authors:** Liusha Dong

**Affiliations:** Yangtze University, JingZhou 434020, China

## Abstract

Music and dance videos have been popular among researchers in recent years. Music is one of the most important forms of human communication; it carries a wealth of emotional information, and it is studied using computer tools. In the feature engineering process, most present machine learning approaches suffer from information loss or insufficient extracted features despite the relevance of computer interface and multimedia technologies in sound and music matching tasks. Multifeature fusion is widely utilized in education, aerospace, intelligent transportation, biomedicine, and other fields, and it plays a critical part in how humans get information. In this research, we offer an effective simulation method for matching dance technique movements with music based on multifeature fusion. The initial step is to use music beat extraction theory to segment the synchronized dance movements and music data, then locate mutation points in the music, and dynamically update the pheromones based on the merits of the dance motions. The audio feature sequence is obtained by extracting audio features from the dancing video's accompanying music. Then, we combine the two sequences to create an entropy value sequence based on audio variations. By comparing the consistency of several approaches for optimizing dance movement simulation trials, the optimized simulation method described in this research has an average consistency of 87%, indicating a high consistency. As a result, even though the background and the subject are readily confused, the algorithm in this research can keep a consistent recognition rate for more complicated dance background music, and the approach in this study can still guarantee a certain accuracy rate.

## 1. Introduction

The most common form is that the dance form evolves in response to the music [1]. Music theme information is communicated through a variety of dance expressions. Dance action matching technology in music arrangement [2] is the process of determining the shape of dance works based on the music style. Effective dance video clip retrieval can assist dance teachers in organizing dance and supporting dance teaching activities [3]. The emotional expression of dancers' works is intimately linked to musical comparison [4]. The dance team's variable or scattered arrangement and creation are similarly difficult to distinguish from the music's production and design [5]. Music is one of the most essential forms of auditory data in multimedia. Computers have carefully studied music as a strong analytical tool in today's digital music era, which has become an unavoidable trend.

In the field of computer vision research [6–8], optimization simulation is currently a highly difficult problem. Its purpose is to analyze dance video data utilizing image processing [9, 10], classification [11], and recognition technology to distinguish motions. With tens of thousands of new songs released each year and the rapid emergence of millions of digital songs that were previously unclassified, existing matching approaches are unable to keep up with the changing times. Because real-world human behavior is based on three-dimensional space, three-dimensional information is critical for music matching optimization simulation. However, extracting 3D information about the human body from RGB dancing photos is difficult. To gather 3D information about the human body, some traditional methods use a depth camera or a laser scanner. The development of matching optimization simulation has been considerably aided by research into human behavior recognition technologies based on artificial intelligence [12] and computer vision. It takes a series of keyframes from a dancing video sequence, generalizes the original video content from high-level semantic information to low-level visual features, and retrieves the original video content using the keyframes as the index, which has a direct impact on video quantity and quality. Final search results in efficiency and accuracy [13].

By annotating the written description of each video frame and matching query keywords with annotations, the multifeature fusion completes the video search [14]. This method begins by incorporating picture band decomposition theory, extracting low-frequency grass-roots information and high-frequency detail information from the dance, and then mapping the corrected grass-roots image. It incorporates multiple functions such as speech, motion, face recognition, and others in a new way, collects diverse human body movements using RGB and infrared cameras, analyzes and recognizes them, and enables intelligent human-computer interaction [15]. It has been discovered that the multifeature fusion of dance and music matching optimization simulation approach may not only aid dance experts assess dance videos but can also be used for teaching, cultural heritage protection, and excavation. The following are the study's unique features: (1) because too many repetitive dance moves in dance motions reduce the retrieval rate, this research provides a method for extracting crucial frames from music and dance videos. (2) In order to improve the classification effect of multimodal features, a multifeature fusion-based optimization simulation method for matching dance and music is proposed, with the goal of transforming low-level audio features into a bag-of-words model that is unified to the lyric text regardless of time or frequency domain. (3) In this study, a multifeature fusion strategy is utilized to learn the implied links between higher-order features recovered by the feature encoding network, allowing for early detection of information interactions between distinct features.

The research framework of this study consists of five major parts, which are organized as follows:

The first part of this study introduces the background and significance of the research and then describes the main work of this study. The second part introduces the work related to the optimal simulation of dance movement and music matching, and multifeature fusion. The third part of the study introduces the design methods of music and dance movement feature extraction and multifeature fusion dance-music matching simulation, so that the readers of this study can have a more comprehensive understanding of the multifeature fusion-based dance-music matching simulation method. The fourth part is the core of the thesis, which completes the description of the multifeature fusion-based optimization simulation analysis from two aspects: optimization simulation and multifeature fusion of dance and music. The last part of the study is the summary of the whole work.

## 2. Related Work

### 2.1. Optimization Simulation of Match between Dance and Music

Music is a kind of artistic expression that is more powerful than images but less so than words. Dance, on this premise, transforms the rich information of dance images buried in music into rich three-dimensional and multidimensional visual images, presenting the meaning of dance to its fullest extent. The significance of music emotion analysis can be seen in the following ways: the study ideas of the music emotion model can be applied to artificial intelligence in emotion recognition, and this research can also be applied to other domains of pattern recognition. Domestication technology and intelligent human-computer interaction have advanced rapidly. The analysis of these music and dance videos is performed using matching optimization simulation, and organically related music and dance action segments are obtained, which not only reduces the work intensity of dance professionals but also facilitates the retrieval of music and dance video data and dance arrangement automation.

Zhou and Zhang developed an application software to improve the content-based matching function on the Internet and make the matching or optimization of music and dance more intelligent [16]. Hong et al. proposed an optimization method based on genetic theory to match the technical movements of dance and music. This method first determines the music style, obtains the basic style characteristics of music and dance, and then analyzes the correlation between the basic characteristics of music and dance to remove the repeated feature pairs [17]. Sun and Ruan used the depth and bone information obtained by the camera for dance action recognition [18]. The recognition accuracy is improved by using the information obtained from the offline data set, including RGB information and available depth and bone information. Ng et al. proposed an optimization method based on machine learning to match dance technical movements and music in music arrangement [19]. First, combined with machine learning theory, this method constructs the mapping relationship between dance action and music based on historical sample data set and obtains the evaluation function of the harmonious relationship between dance action and music. Wang et al. proposed a method to quickly and accurately predict the 3D position of dance movements in a single depth image without using time information [20].

### 2.2. Research on Multifeature Fusion

In the human perception of music, a music category refers to a group of songs that usually feel the same interpretation. Music genres provide important emotional descriptions and are used to classify music. In recent years, many domestic and foreign scientific research institutes and relevant scholars are committed to the research of dance movement recognition, which has made great contributions to the development of movement recognition research. However, how to classify dance movements and music in the music genre classification system is an arduous task.

Zhang and Zhao proposed an optimization method for matching dance technique movements to music based on greedy theory [21]. The method now adapts a given dance movement and that movement to the beat of the music, and then performs music-dance movement matching based on this. According to Pandeya and Lee motion recognition based on static RGB image features, in videos dealing with complex backgrounds, static features are susceptible to factors such as background, illumination, and human motion, making feature extraction difficult [22]. Huang et al. focused on dynamic scene understanding, target tracking, and motion recognition through multifeature fusion and successfully applied it to applications such as real-time surveillance, teleconferencing, and intelligent robot navigation [23]. López-Ortega proposed an optimal matching method for multifeature fusion images based on correction and balancing techniques in dance [24]. The method first maps the luminance of each pixel in the dance correction and balance technique image to the luminance range that can be output by the display device according to a one-to-one correspondence. Roy et al. developed an intelligent video surveillance system based on multifeature fusion that overcomes the interference of scene illumination changes and can automatically detect music in the video with the function of automatically matching the dance [25].

The dance competition is not only a competition for dancers' skills but also a competition for general arts other than dance, such as music creation, theme script, and stage art. As an important part of dance, dance music is unparalleled in dance works.

## 3. Optimization Simulation Method of Dance and Music Matching Based on Multifeature Fusion

### 3.1. Feature Extraction of Music and Dance Movements

The variability of dance movements and too many overlapping movements leads to major problems in extracting movement features [26]. The movements of music and dance videos are complex, changeable, and repetitive, which makes it difficult to analyze and identify dance movements [27]. The artistic form of music is stronger than abstraction and weaker than an image, but its rigid organizational logic, artistic structure, and rich symbolic meaning strengthen people's thoughts and connect and synthesize metaphors into moving sounds [28]. On this basis, a genetic algorithm is used to train the corresponding relationship of different music and dance movements, and its accuracy is taken as the fitness function to obtain the optimal music and dance movement matching. People are greatly inspired by the research in the field of art and music psychology. The analysis model of music emotion perception is shown in Figure 1.

First, in the process of dance action matching and optimization in music arrangement, the synchronized dance action and music data are segmented through music beat extraction theory to obtain multiple short action music fragment combinations. After calculating the entropy value of each image in the image sequence, the entropy value corresponding to the current frame is compared with the previous frame. If it is greater than the threshold, it is considered as a keyframe. The following formula is often used to calculate the entropy between samples. The smaller the entropy, the greater the similarity between samples. For an *n* dimensional space, the Minkowski distance between point *X* and point *Y* can be expressed as follows:

(1) $$\begin{array}{c} di\;s\left(X,Y\right)=\sqrt[{p}]{\sum_{i=1}^{n}{\left|x_{i}-y_{i}\right|}^{p},i=1,2,...,n}, \end{array}$$

where *x*_*i*_ is the *i* dimensional characteristic data of point *X* and y_*i*_ is the*i* dimensional characteristic data of point *Y*.

Using the keyframe sequence as input, the RGB image information of the keyframes is input to the spatial convolutional neural network to extract the video shape information and the optical flow information of the keyframes and adjacent frames, which is used to extract the temporal convolutional network motion information of the video frames. Therefore, in this study, each joint point of the image is assigned a motion contribution weight, and the joint contribution weight formula of the feature vector can be expressed as follows:

(2) $$\begin{array}{c} \text{dis}\left(x^{\left(m\right)},x^{\left(n\right)}\right)=\sqrt{\sum_{i=1}^{N}\omega_{i}{\left(x_{ix}^{\left(m\right)}-x_{ix}^{\left(n\right)}\right)}^{2}+{\left(x_{iy}^{\left(m\right)}-x_{iy}^{\left(n\right)}\right)}^{2}}. \end{array}$$

Before the comparison, in order to select more representative features and reduce the computational complexity, the CHI feature selection method based on the difference mentioned above is used to select features for both audio words and text words. Generally, the feature extraction process is shown in Figure 2.

Second, the transition point of music is detected, the beat prediction position obtained in each stage is aligned, the correlation coefficient between dance action and music part is calculated, and the dance action matching optimization objective function is obtained. The dance action is represented by the dispersion of different coordinate positions in the whole video. The more active the action is, the higher the dispersion degree is. The dispersion degree of dance action *i* is measured by the variance of coordinates:

(3) $$\begin{array}{c} \sigma_{i}^{2}=\frac{\sum_{f=0}^{n}{\left(x_{i}^{\left(f\right)}-x_{i}\right)}^{2}+{\left(y_{i}^{\left(f\right)}-y_{i}\right)}^{2}}{n}. \end{array}$$

Here, *x*_*i*_^(*f*)^, *x*_*i*_ are the abscissa and ordinate positions of joint point *i* in frame *f*, *x*_*i*_, *y*_*i*_ are the average abscissa and ordinate positions in the whole video sequence, and *n* is the video frames.

Then, the motion contribution weight of joint point *i* can be expressed as follows:

(4) $$\begin{array}{c} \omega_{i}=\frac{\sigma_{i}^{2}}{\sum_{k=0}^{n}\sigma_{k}^{2}}. \end{array}$$

The duration of the dance video, the number of frames in the image, and the frame rate of the video are all known during these audio and dance movements, and interval operations are performed using standard deviations, corresponding to audio and audio values computed once per second. Entropy value sequences and functions are combined [29]. The contrast and visual quality of the image are increased by mapping pixels concentrated in several grayscales to other grayscales and distributing them uniformly by dividing the color gamut point by point by the chromaticity priority of the standard layer image [30].

Finally, to achieve dance action matching in music arrangement, all music and dance action parts of the music arrangement are adaptively adjusted to pheromone fluctuation factors according to pheromone concentration, and pheromones are dynamically updated according to the optimal solution of dance action matching. The order of entropy values is calculated after feature fusion. In comparison, the difference in entropy values between two adjacent frames is not utilized as a benchmark for determining keyframes, but instead, it is determined by comparing this value with the threshold using the following formula:

(5) $$\begin{array}{c} \text{V}=\frac{\left|H_{\text{current}}-H_{\text{key}}\right|}{H_{\text{key}}}. \end{array}$$

Here, *H*_*current*_ is the entropy value of current frame and *H*_*key*_ is the entropy of the current keyframe.

For the skeleton 3D coordinate data in each frame of the video sequence, k frame is randomly selected as the sample center, and then the 30 3D coordinate data in k extracted at last are unchanged or less than a certain threshold through iteration in turn by using the above algorithm.

### 3.2. Specific Design of Multifeature Fusion Dance and Music Matching Optimization Simulation

In the first mock exam of video, there are many modes in its content, such as appearance, optical flow, and depth. These modes complement each other, convey important information, and integrate these modes, which can effectively solve the problem of insufficient expression of single modal video information. The distance between the keyframe sequence *KF* and the original video sequence set *F* can be expressed by the maximum semi Hausdorff, which is defined as follows:

(6) $$\begin{array}{c} D=\left(F,KF\right)=\max\left\{D\left(F_{i},KF\right)|i=1,2,\ldots ,N\right\}. \end{array}$$

Music in a narrow sense refers to the basic elements of music sound, including pitch, length, intensity, and timbre. These basic elements combine to form the “formal elements” of common music. After extracting low-level features from audio's auditory and visual features, we use feature coding network to study the low-level features to obtain high-level features. Emotion recognition presents a hierarchical feature, as shown in Figure 3.

Because music genres are often distributed in local and repeated audio clips, if the music is divided into segments that are too short, it will be difficult to reflect the relationship between local characteristics. The specific design method of multifeature fusion music recognition method is shown below.

First, the optical flow information in the video is extracted by the denseflow software, and the video is divided into frames. Recall (*R*) is used to measure the missing detection of extracted keyframes and can be expressed as follows:

(7) $$\begin{array}{c} R=\frac{N_{c}}{N_{c}+N_{m}}\times 100\%. \end{array}$$

Here, *N*_*c*_ is the number of keyframes correctly extracted from the extracted results and *N*_*m*_ is the number of missed keyframes.

The open pose posture estimation tool is used to extract the coordinate information of human joints in the image and normalize it. First, the collected music data are divided, and the movement segments are connected and constructed in the dance movement database, so as to obtain the basic features of historical music and dance movements, extract some feature pairs by correlation analysis, and calculate the gender coefficient by the correlation between music and dance features. In order to avoid the situation that the weight tends to be long text, which is not conducive to short text, this study normalizes the weight of the calculated feature words, and the formula is as follows:

(8) $$\begin{array}{c} W\left(t,d\right)=\frac{1+\;\log_{2}\;tf\left(t,d\right)\times \;\log_{2}\left(N/n_{l}\right)}{\sqrt{-\sum_{t\in d}\left[\left(1+\;\log_{2}\;tf\left(t,d\right)\times \;\log_{2}\left(N/n_{l}\right)\right)\right]}}. \end{array}$$

Here, *W*(*t*, *d*) is the weight, *tf*(*t*, *d*) is the frequency, *N* is the total number of all videos in the training set, and *n*_*t*_ is the number of documents, in which the feature word t appears.

In the actual work process, if the length of the lens and the complexity of the video content under the lens are not considered, if the lens is too long, it is difficult to summarize the content of the lens with only a few music clips. Therefore, relevant features are extracted from the original data according to the needs and analyzed and processed in combination with the differences of various feature information. The difference here is defined as follows:

(9) $$\begin{array}{c} \Delta \;di\;s\left(w\right)=\frac{abs\left(chi_{i}-chi_{j}\right)}{\sqrt{\max\left(chi_{i},chi_{j}\right)}}. \end{array}$$

Second, we constructed temporal and spatial convolutional network models based on the Res Net152 structure, respectively, and then fine-tuned the dual-stream network model by migration learning to obtain high-level semantic features, image functions, and optical stream functions of RGB. In this system, audio features and lyric features are fused at the feature level, and the fusion is done in a linked manner. That is, the features of the two modes are directly linked to form a new feature vector. Unlike semi-infinite linear programming, it exploits the smoothing property of the objective function and uses gradient descent to update the kernel function weights. The kernel function weights are given by the following equation:

(10) $$\begin{array}{c} D_{m}=\left\{\begin{array}{c} 1,\left(\text{if }dm=1,\text{and}\frac{\partial J}{\partial d_{m}}-\frac{\partial J}{\partial d_{\mu }}>0\right)\\ -\frac{\partial J}{\partial d_{m}}+\frac{\partial J}{\partial d_{\mu }}\left(i\text{f }dm\;>1,\text{and }m\neq \mu \right)\\ \sum_{i=1}\frac{\partial J}{\partial d_{v}}-\frac{\partial J}{\partial d_{\mu }}\left(if\;m=\mu \right) \end{array}\right.. \end{array}$$

Here, *D*_*m*_ is the direction of gradient descent.

To keep the input sample size sufficient and increase the number of input samples, the original audio stream is separated into continuous segments. The trajectories created by SIFT matching between video frames are one type, while the trajectories obtained by optical flow tracking sampling points are the other. The sampling sites are sampled near each sift point. Finally, we construct a spatiotemporal graph convolutional neural network model based on the graph convolutional neural network structure to capture the spatial information of the joint points in the time series. Then, based on the extracted audio sentiment features, these features are used to obtain a pixel-value representation of the lyrics based on the codebook. The new pixel value is considered as a background pixel when the nearest Gaussian distribution belongs to any of the above B Gaussian distributions; otherwise, it is a foreground pixel. Then, a sector template with a circular angle of 70° is rotated and slid in a circular area to obtain the vector formed by the sum of the Harr responses in each sliding window, and the direction corresponding to the maximum of the sum of the sums is chosen as the reference direction of the feature.

## 4. Simulation Analysis of Matching Optimization Based on Multifeature Fusion

### 4.1. Optimization Analysis

When we appreciate dance (especially the artistic dance carefully created by choreographers), music and its melody, harmony, rhythm, mode, and texture are indispensable components of dance works. In the process of music and dance movement matching optimization, based on the objective function of dance movement matching optimization, combined with the optimization simulation theory, the objective function is optimized. The concentration adaptively adjusts the pheromone volatilization factor, dynamically updates the pheromone according to the advantages and disadvantages of the optimal dance action matching scheme, and completes the dance action matching optimization in music choreography. Since the features extracted here are exactly the same as those in the single-mode music emotion recognition based on audio, the main factor to judge whether the two clips are similar is the feature factor, which is the feature value video obtained by matching the information. It is the principal component to measure whether two things are consistent with one result. Therefore, the characteristic factors should occupy a high weight. The accuracy of video clips in the two dance data sets under different weights is shown in Figure 4.

First, we create a sliding window containing many pixels in the window and use the median of all these pixels as the new value for the center of the window. Viewing a band in this window, the harmonic content remains fairly constant, while the shock structure is shown as a peak. Low-level music features usually use statistical function variables to summarize the variance or central tendency in the music. Among them, the boundary direction histogram is a boundary-based shape analysis method that is independent of the size and location of the image object, simple to compute, and can better describe the shape of the object boundary. In this section, the Mel spectrogram of the dataset is used as an input to select the appropriate size of music segments and the number of heads in the feature encoding network, and the results are shown in Figure 5.

Second, it sorts the gray values of all pixels in the window. After sorting, the median of the array is taken as the new value of the gray value of the central pixel of the window. According to the comparison results between the ratio of the nearest distance and the next nearest distance and the threshold, a pair of matching points is accepted, then one-way matching is completed, whether to obtain a group of candidate matching pairs is judged, and the same method of using the matching points of the next frame is used to inverse match with the previous frame to obtain a pair of inverse matching feature points. Because it is difficult to describe and measure an image frame accurately and comprehensively by relying on only one image feature, it is necessary to integrate several different image features to measure the similarity in order to describe the original image content more comprehensively and accurately. This study compares the different *λ* values that affect the experiment. The results show that the best test accuracy can be obtained when the value of *λ* is set to 0.05. The influence of self-attention mechanism and net VLAD on a feature coding network is shown in Figure 6.

Finally, the directional gradient histogram feature used to describe the dance movement information is extracted from the image. Features are described as the boundary direction histogram, and texture features are described as wavelet transform containing various image features.

This is because the method in this study first incorporates music beat extraction theory to segment the synchronized dance movement and music data to obtain multiple short movement-music fragment combinations and calculate the correlation between the dance movement-music fragments. It is used to obtain the optimal objective function for dance movement matching, which improves the degree of dance movement-music matching in the music choreography performed by the method of this study.

### 4.2. Multifeature Fusion Analysis of Dance and Music

The smallest unit of any fully structured music is a part. The phrases and parts in a part are the internal building blocks of the structural unit. Similarly, the features of dance images provide other information for motion recognition, and image features provide appearance information closely related to the human movement in the image in the process of motion recognition. The comprehensive effectiveness of this method needs to be verified by simulation. The experimental data are from the dance action capture database provided by Carnegie Mellon University Laboratory, and the length of each music segment is about 5 seconds. Using the methods of this study and references [17] and [19], the optimization experiment of dance action matching in music choreography is carried out, and the matching degrees (%) of the three methods are compared.  Figure 7 shows the comparison results of dance movements in music arrangement.

The results show that the average matching degree between the optimized simulation methods in this study is 87%, and the matching degree is very high. This is mainly because the method in this study first detects the transition point of a music segment, aligns the beat prediction position obtained in each stage, and adaptively adjusts the pheromone fluctuation factor according to the pheromone concentration of all music dance motion segments. The music arrangement uses the method of this study to match the dance movements well.

The calculation procedure is to use the *k* vectors clustered out in each video sequence about the sample centers of 3D joint node positions, the clustering centers of the joints in each vector, and the coordinates of the corresponding 3D joints in each frame of the video sequence to calculate the Euclidean distance, respectively. The appearance information of objects in an image can be well described by the direction of gradients or edges, and the method generates descriptors by calculating the statistical information of local image gradient directions. Two images can be generated by using a median filter to filter in the horizontal and vertical directions of the magnitude spectrogram of the descriptor. If the median filter is applied at the frequency, the shock events are enhanced and the harmonic components are suppressed. The best combination of features is input to the meta-CNN and the training process is visualized on the model GTZAN and Extended Ballroom datasets. The results are shown in Figure 8.

Second, in the training process, the feature pyramid network (FPN) extracts features and returns to the key points of human skeleton, and the simple key points will be basically completed in the FPN stage. The detailed network structure of FPN is listed in Table 1.

Multicore learning can be understood as having great interpretability when learning the weighted convex combination of several cores, and the weight coefficient is crucial for extracting features from different modes. It is possible that such a probability value is zero. To avoid the occurrence of zero probability, it is a common practice to apply various data smoothing procedures. A pixel with a significant difference value in two orthogonal directions is particularly unique and ideal for tracking, even if it is on an edge. As a result, the RGB picture data recovered from the keyframe, as well as the stacked optical flow generated by the keyframe and its surrounding 10 frames, are fed into the spatial and temporal convolution networks for testing. The results are listed in Table 2.

Finally, the strong and weak edges and details of each layer are separated by limiting the number of strong edges, then the layered mapping function is constructed for each layer, and point-by-point mapping is performed for each layer by enhancing the details of each layer and the contrast of the weak edges and keeping the strong edges, thus realizing the remapping process for each layer. The video frame with the largest *C* value is calculated, the index of the frame with that *C* value is obtained, and finally, the keyframes are sorted by index value, and if the number of indexes is the same, the keyframes are determined based on the sum of the calculated distance between the nodes in the frame and the nodes corresponding to the clustering center, and the one with the smallest sum is the keyframe. Thus, the edge features of each image of a video frame are accumulated in a single image, and finally, the directional gradient histogram features are extracted from the image of the accumulated edge features.

## 5. Conclusions

Unique or expressive rhythms, such as strength, weight, and melody, are primarily used to define the integration of music and dance. Music sentiment analysis, such as music sentiment expression models, music review feature identification, emotional music classification, and emotional music search, is a hot trend in artificial intelligence. Music and dance matching is crucial in music discovery and can be used to manage and tag music content on websites and device music engines. On the basis of multifeature fusion, a strategy is given for optimizing dance technology movement and music matching simulation. By obtaining optimal performance on a dataset, multifeature fusion illustrates a good application case. The multifeature fusion-based dance and music matching optimization simulation approach, which includes feature extraction of music and dance movements, is described in this work. The dance music multifeature fusion and multifeature fusion-based matching optimization simulations are thoroughly examined. This aggressive and comprehensive matching approach is more universal and scalable, and it can give a platform for additional distinct songs and dances besides chime music and dance. In this way, the same cultural isomorphism, emotional isomorphism, affective isomorphism, and imagery synthesis of music and dance matching can both express the music's sensual characteristics and reach the audience's mind. Music expresses emotion, while music ultimately reproduces the form of space through dance, ultimately creating an audience through audio-visual fusion.

## Figures and Tables

**Figure 1:** Analysis model of music emotion recognition.

**Figure 2:** Feature extraction process diagram.

**Figure 3:** Hierarchical characteristics of music emotional cognition.

**Figure 4:** Accuracy of video clips in two dance datasets under different weights.

**Figure 5:** Test accuracy of music segment and feature coding network.

**Figure 6:** Influence of self-attention mechanism and net VLAD on feature coding network.

**Figure 7:** Comparison chart of matching degree of different methods of dance movements.

**Figure 8:** Training results.

**Table 1:** Detailed structure of FPN network.

Type of layer	Step size and number of fills	Output size	Nuclear size
Conv1D	3.0	(10, *b*, 84)	(34, 969)

ReLU	2.5	(28, 76, 32)	(27, 1004)

Dense	1.8	(27, 47, 44)	(29, 1863)

Maxpooling1D	2.2	(43, 34, 38)	(63, 548)

**Table 2:** Accuracy of different keyframes on ufc101 split1.

Number of keyframes	10	20	30
Accuracy (%)	44.8	52.9	89.8
Average consumption time (s)	3.6	4.2	2.1

## Data Availability

The data used to support the findings of this study are available from the corresponding author upon request.
